RETRACTED

# Analysis on the Clinical Effect of High-Dose Glucocorticoids Combined with Immunosuppressants on Patients with Myasthenia Gravis Undergoing Video-Assisted Thoracoscopic Surgery

**DOI:** 10.1155/2021/5854056

**Published:** 2021-12-06

**Authors:** Pei Liu, Haoyue Wang, Jiejie Hu, Xiaobin Zhai, Zhaoming Ge

**Affiliations:** Department of Neurology, Lanzhou University Second Hospital, Lanzhou, 730030 Gansu Province, China

## Abstract

**Objective:**

The purpose of the study was to investigate the clinical effect of high-dose glucocorticoids (GCS) combined with immunosuppressants on the treatment of myasthenia gravis (MG) with video-assisted thoracoscopic surgery (VATS).

**Methods:**

A total of 106 MG patients admitted to the neurology department of our hospital from February 2016 to February 2020 were selected as the study subjects and divided into experimental group (*n* = 53) and control group (*n* = 53). The patients in the control group underwent VATS, while the patients in the experimental group were treated with high-dose GCS combined with immunosuppressants on the basis of VATS treatment. The clinical efficacy of different MG treatment methods was analyzed.

**Results:**

No significant differences were observed in visual analogue score (VAS) at T1 between the two groups (*P* > 0.05), while VAS scores at T2, T3, and T4 in the experimental group were significantly lower than those in the control group (*P* < 0.001). In the experimental group, the overall response rate was significantly higher than the control group (*P* < 0.05). Cytotoxic T-lymphocyte-associated protein 4 (CTLA4) level in regulatory T (Treg) cells in experimental groups after treatment was significantly higher, compared to that in before treatment and the control group (*P* < 0.05). Similar results of each quantitative MG score were displayed in both groups after treatment, compared to before treatment and the control group (*P* < 0.05). Clinical performance of patients with lower incidence of adverse reactions in the experimental groups after treatment was significantly higher than those in the control group (*P* < 0.001).

**Conclusion:**

GCS combined with immunosuppressants can effectively relieve patients' clinical symptoms and improve their quality of life, with significant clinical efficacy and high safety, which is worthy of application and promotion.

## 1. Introduction

Myasthenia gravis (MG), as an immune disease in neurology, refers to weak contraction in skeletal muscles caused by impairment of neuromuscular transmission. The clinical hallmark of MG consists of fluctuating fatigability and weakness affecting ocular, bulbar, and (proximal) limb skeletal muscle groups. A pragmatic clinical classification distinguishes pure ocular myasthenia from generalized myasthenia with mild, moderate, and severe manifestation. Ocular myasthenia exclusively affects the outer ocular muscles including the M. levator palpebrae and presents with ptosis and double vision. Ptosis and double vision may be transient, fluctuating, or progressive during the day. Only 10–20% of patients show muscle fatigability and weakness persistently restricted to the outer ocular muscles. The majority of patients proceed to generalized muscle fatigability and weakness within 24 months after the disease onset [1, 2]. Investigations have found that MG, which has affected 730000 patients across the whole world, can occur at any age and be specifically divided into generalized and ocular types, with higher prevalence rate in women than in men [3]. At present, the top priority for MG treatment is drug therapy, in which glucocorticoids (GCS) and immunosuppressants have been widely used, as GCS can effectively improve thymus immune function, inhibit germinal center formation, and promote the secretion of acetylcholine at the neuromuscular junction, thus greatly relieving clinical symptoms [4, 5]. However, clinical practice confirms that long-term implementation of drug therapy can contribute to multiple complications, hence increasing the difficulty of treatment. Some scholars have pointed out that immunosuppressants combined with GCS can greatly shorten treatment time and effectively avoid the side effect caused by the long-term use of hormones, thus exerting the synergistic effect of drugs and improving therapeutic effect [6]. As a minimally invasive treatment method, video-assisted thoracoscopic surgery (VATS), which is performed with the assistance of high-definition video-assisted photographic technology and high-tech equipment, with the advantages of less trauma and obvious clinical efficacy, has been widely applied in thoracic surgery [7]. This study provides more evidence for MG treatment by further investigating the clinical effect of high-dose GCS combined with immunosuppressants on MG treatment with VATS, and the study is reported as follows.

RETRACTED

## 2. Materials and Methods

### 2.1. General Information

A total of 106 MG patients admitted to the neurology department of our hospital from February 2016 to February 2020 were selected as the study subjects and divided into experimental group (*n* = 53) and control group (*n* = 53), according to the number table method. In the experimental group, there were 28 males and 25 females, with the average age of 46.52 ± 5.83 years old, average course of disease of 5.63 ± 1.24 months, and average body mass index (BMI) of 21.43 ± 1.22 kg/m^2^, including 24 patients in the acute phase and 29 in the remission phase, while in the control group, there were 27 males and 26 females, with the average age of 46.54 ± 5.81 years old, average course of disease of 5.66 ± 1.26 months, and average BMI of 21.46 ± 1.23 kg/m^2^, including 26 patients in the acute phase and 27 in the remission phase, with comparability.

This study was approved by the Hospital Ethics Committee, and patients and their family members were informed of the purpose and processes of this study and signed the informed consent.

### 2.2. Inclusion Criteria

Patients diagnosed with MG by internationally recognized diagnostic criteria, not restricted in age, gender, ethnicity, race, and disease stage, met the diagnostic criteria for MG, were treated with VATS, and had complete clinical data, were included.

### 2.3. Exclusion Criteria

Patients who had malignant tumors, had other immune system diseases, had surgical contraindications or were in lactation period, had mental and other cognitive disorders, and had severe cardiovascular diseases, mental illnesses, etc., will be excluded.

### 2.4. Methods

In the control group, the patients, after taking supine positions, underwent VATS treatment. During surgery, an approximately 3 cm incision made in the 3rd intercostal space of anterior axillary line on the posterior border of the right pectoralis major muscle was taken as the main operating hole, and an approximately 1.5 cm incision made in the 5 h intercostal space of midaxillary line was taken as the observation hole. Subsequently, after CO_2_ pneumothorax was established with appropriate pressure, the medistinal pleura was cut vertically along superior vena cava and anterior phrenic nerve, and then, the pleura was cut parallelly along sternum and posterior arteries and veins in thoracic cage, until the thymus was completely removed [8, 9].

On the basis of the treatment in the control group, the patients in the experimental group were treated with high-dose GCS combined with immunosuppressants. The intravenous injection of prednisolone (State Food and Drug Administration approval number: H33020824; manufacturer: Huazhong Pharmaceutical Co., Ltd.; specification: 5 ml: 0.125 g) was performed, 1000 mg/d × 3d, and the dosage was halved every 3 d until the 27th d. At the same time, the patients should take ciclosporin (State Food and Drug Administration approval number: H10960123; manufacturer: Hangzhou Zhongmei Huadong Pharmaceutical Co., Ltd.; specification: 50 mg∗50 s) orally at the dose of 1 mg/(kg · d) for the first 3 d, 2 mg/(kg · d) for 4-6 d, 4 mg/(kg · d) for 7-10 d, and 4 mg/(kg · d) for maintenance, and they also should take mycophenolate mofetil (State Food and Drug Administration approval number: H20031277; manufacturer: Shanghai Roche Pharmaceutical Co., Ltd.; specification: 0.5 g∗20 s) orally, at the dose of 0.5 g/d for the first 3 d, 1 g/d for the first 4-6 d, 1.5 g/d for the first 7-10 d, and 1.5 g/d for maintenance. Additionally, intravenous drip of 10-15 mg/kg cyclophosphamide (State Food and Drug Administration approval number: H32024654; manufacturer: Jiangsu Shengdi Pharmaceutical Co., Ltd.; specification: 0.2 g × 1 vial/box) was also performed, once a week, with the total dose of 10 g.

RETRACTED

### 2.5. Evaluation Indexes

VAS score [10] was adopted to evaluate the degree of limb pain at different time points in the two groups, with the total score of 10 points, and higher scores indicated severer pain. The time points at 1 d, 3 d, 7 d, and 14 d after surgery were set as T1, T2, T3, and T4, respectively.

Quantitative MG score scale [11] was adopted to evaluate patients' limb recovery before and after treatment, with five scoring items and each giving a total score of 10 out of 50, and higher scores indicated better limb recovery.

According to the results of quantitative MG score scale, the treatment effect was categorized as 5 levels, which were summarized as follows. Recovery referred to that patients' total MG score decreased by more than or equal to 95%, compared with the score before treatment; the markedly effective referred to that patients' MG score decreased by 80-94%; the improved referred to that patients' MG score decreased by 60-79%; the effective referred to that patients' MG score decreased by 30-59; the ineffective referred to that patients' MG score decreased by less than or equal to 29%. The total effective rate = recovery rate + markedly effective rate + improved rate + effective rate.

5 ml of fasting venous blood samples were collected from patients in both groups before and after treatment, and the CTLA4 levels in Treg cells were measured by Attune NxT flow cytometer (manufacturer: Beijing Heros Technology Co., Ltd.).

Quality of life of the patients in both groups after treatment was evaluated by the postoperative quality of life scale for MG patients, which was made in our department, with five items in total and each scoring 20 points, and higher scores indicated better quality of life.

The incidence of adverse reactions of the patients was recorded and compared between the two groups.

### 2.6. Statistical Analysis

All the data were processed for statistical analysis by SPSS21.0 software, and GraphPad Prism 7 (GraphPad Software, San Diego, USA) was used to draw the pictures of the data. Measurement data were expressed by ($\bar{\text{x}}\pm \text{s}$) and tested by *t*-test. Enumeration data were expressed as [*n* (%)] and tested by *χ*^2^ test. The differences had statistical significance when *P* < 0.05.

RETRACTED

## 3. Results

### 3.1. Comparison of VAS Scores at Different Time Points after Surgery between the Two Groups

There were no significant differences in VAS scores between the two groups at T1 (*P* > 0.05), and the VAS scores in the experimental group at T2, T3, and T4 were significantly lower than those in the control group (*P* < 0.05), as shown in Figure 1.

### 3.2. Comparison of Therapeutic Effect between the Two Groups

The overall response rate in the experimental group was significantly higher than that in the control group (*P* < 0.05), as shown in Table 1.

### 3.3. Comparison of CTLA4 Levels in Treg Cells before and after Treatment between the Two Groups

The CTLA4 levels in Treg cells in both groups after treatment were significantly higher than those before treatment (*P* < 0.05), and the CTLA4 levels in Treg cells in the experimental group after treatment were significantly higher than those in the control group (*P* < 0.05), as shown in Figure 2.

### 3.4. Comparison of Quantitative MG Scores before and after Treatment between the Two Groups

Each quantitative MG score in the two groups after treatment was significantly higher than that before treatment (*P* < 0.05), and each quantitative MG score in the experimental group after treatment was significantly higher than that in the control group (*P* < 0.05), as shown in Table 2.

### 3.5. Comparison of Quality of Life Scores after Treatment between the Two Groups

After treatment, the limb function, linguistic function, emotional function, vitality, and cognitive function of the patients in the experimental group were all significantly higher than those in the control group (*P* < 0.05), as shown in Table 3.

### 3.6. Comparison of Incidence of Adverse Reactions between the Two Groups

The incidence of adverse reactions in the experimental group after treatment was significantly lower than that in the control group (*P* < 0.05), as shown in Table 4.

## 4. Discussion

MG is an autoimmune antibody-mediated disorder of neuromuscular synaptic transmission. In early stage, patients generally present with weakness of limbs, and with the progress of this disease, they may suffer from dysphagia, low spirits, and even breathing difficulties. MG may either occur as an autoimmune disease with distinct immunogenetic characteristics or as a paraneoplastic syndrome associated with tumors of the thymus. At present, the medical community has not found the specific pathogenesis of MG and has presumed that it may be associated with infection factors, environmental factors, etc. [12–14]. Immunosuppressants combined with GCS is effective for some MG patients, except for a minority of patients. GCS, as a common treatment method for MG including prednisolone, betamethasone, and dexamethasone, plays a key regulatory role in body growth, metabolism, and immune function, and is the most important regulatory hormone in stress response, which can effectively inhibit patients' immune inflammatory response and pathological immune response; however, it is found that long-term adoption also comes with toxic and side effect [15–17]. In addition, long-term administration of hormone drugs can result in adrenal cortex function decline, osteoporosis, femoral head necrosis, etc. Immunosuppressants can inhibit the proliferation of cells involved in the immune response and reduce the antibody immune response, thereby relieving patients' clinical symptoms [18, 19].

RETRACTED

VATS, as a minimally invasive surgery which has been widely applied for the treatment of thoracic diseases, can visualize patients' thorax clearly on a television screen through a high-definition camera, so the surgeon can conduct the surgery by viewing a television screen, with the advantages of wide range of lesion resection and high safety [20, 21]. Some studies reveal that the thymusectomy not only removes the thymus but also effectively clears the fat of anterior mediastinum, but VATS is limited by the surgical field during the resection of the fat of anterior mediastinum, so the surgical procedure should be finished by experienced operators [22, 23]. In this study, after the combination therapy was implemented in MG patients, the overall response rate in the experimental group was significantly higher than that in the control group (*P* < 0.05), demonstrating that the combination therapy has significantly better efficacy than VATS alone in relieving myasthenic symptoms and improving prognosis. Treg cells are T cell subsets that negatively regulate immune responses and maintain immune tolerance, and their number and function defects greatly affect the development and progression of MG. CTLA4, as a critical negative regulator of the T-cell response, maps to chromosome 2q33 and is involved in the negative regulation of immune responses [24, 25]. It has been considered a candidate for many autoimmune diseases. Evidence from Caucasians supported a genetic predisposition of CTLA4 to myasthenia gravis (MG). Several variants of CTLA4 have been extensively tested, indicating an overall influence on the susceptibility of several immune-related diseases [24]. In this study, we found that CTLA4 levels in Treg cells in the experimental group were significantly higher than those in the control group (*P* < 0.001). Chandeze et al. [26] have pointed out in their study that after the implementation of VATS combined with short course of high-dose GCS and immunosuppressants in patients with late-onset and severe MG, the CTLA4 levels in Treg cells of the patients who underwent the treatment were (16.42 ± 2.23)%, which were significantly higher than (11.76 ± 2.15)% of the patients who were treated with VATS alone, illustrating that the combination therapy can enhance the Treg cells levels in the peripheral blood of MG patients and improve therapeutic effect.

RETRACTED

In conclusion, the combination therapy can significantly relieve myasthenic symptoms and improve quality of life of patients, with significant therapeutic efficacy and high safety, which is worthy of application and promotion.

## Figures and Tables

**Figure 1:** Comparison of VAS scores at different time points after surgery between the two groups ($\bar{\text{x}}\pm \text{s}$). Note: the abscissa represented T1, T2, T3, and T4, while the ordinate represented VAS score, points. The VAS scores at T1, T2, T3, and T4 in the experimental group were 6.32 ± 0.43 points, 5.17 ± 0.34 points, 3.24 ± 0.28 points, and 1.92 ± 0.23 points, respectively. The VAS scores at T1, T2, T3, and T4 in the control group were 6.35 ± 0.46 points, 5.86 ± 0.32 points, 4.56 ± 0.31 points, and 2.83 ± 0.21 points. ^∗^ indicated that there were significant differences in VAS score at T2 between the two groups (*t* = 10.759, *P* < 0.001). ^∗∗^ indicated that there were significant differences in VAS score at T3 between the two groups (*t* = 23.005, *P* < 0.001). ^∗∗∗^ indicated that there were significant differences in VAS score at T4 between the two groups (*t* = 21.271, *P* < 0.001).

**Figure 2:** Comparison of CTLA4 levels in Treg cells before and after treatment between the two groups ($\bar{\text{x}}\pm \text{s}$). Note: the abscissa represented before and after treatment, while the ordinate represented CTLA4 level in Treg cells. The CTLA4 levels in Treg cells in the experimental group before and after treatment were 9.84 ± 1.53% and 16.59 ± 2.17%, respectively, while those in the control group were 9.89 ± 1.55% and 12.36 ± 2.13%, respectively. ^∗^ indicated that there were significant differences in CTLA4 levels in Treg cells before and after treatment in the experimental group (*t* = 18.508, *P* < 0.001). ^∗∗^ indicated that there were significant differences in CTLA4 levels in Treg cells before and after treatment in the control group (*t* = 6.826, *P* < 0.001); ^∗∗∗^ indicated that there were significant differences in CTLA4 levels in Treg cells after treatment between the two groups (*t* = 10.128, *P* < 0.001).

RETRACTED

**Table 1:** Comparison of therapeutic effect between the two groups [*n* (%)].

Group	*n*	Recovery	Markedly effective	Improved	Effective	Ineffective	Overall response rate
Experimental group	53	7 (13.21%)	23 (43.40%)	16 (30.19%)	5 (9.43%)	2 (3.77%)	96.23% (51/53)
Control group	53	2 (3.77%)	14 (26.42%)	12 (22.64%)	16 (30.19%)	9 (16.98%)	83.02% (44/53)
*χ* ^2^							4.970
*P*							0.026

**Table 2:** Comparison of quantitative MG scores before and after treatment between the two groups ($\bar{\text{x}}\pm \text{s}$, points).

Group	Experimental group (*n* = 53)		Control group (*n* = 53)	
	Before treatment	After treatment	Before treatment	After treatment
Upper limb	3.26 ± 0.42	6.73 ± 0.51	3.28 ± 0.39	4.58 ± 0.49^∗^
Head	2.17 ± 0.24	11.43 ± 0.45	2.19 ± 0.25	7.84 ± 0.42^∗^
Lower limb	3.11 ± 0.24	6.81 ± 0.45	3.09 ± 0.26	4.61 ± 0.48^∗^
Facial muscles	2.63 ± 0.32	7.49 ± 0.36	2.67 ± 0.29	5.02 ± 0.42^∗^
Swallowing	2.04 ± 0.25	8.01 ± 0.33	2.06 ± 0.31	6.04 ± 0.37^∗^
Score	13.21 ± 1.47	40.47 ± 2.10	13.29 ± 1.50	28.09 ± 2.18

Note: each quantitative MG score in the two groups after treatment was significantly higher than that before treatment; ^∗^ indicated the comparison of each quantitative MG score after treatment between the two groups, *P* < 0.05.

**Table 3:** Comparison of quality of life scores after treatment between the two groups ($\bar{\text{x}}\pm \text{s}$, points).

Group	*n*	Limb function	Linguistic function	Emotional function	Vitality	Cognitive function
Experimental group	53	14.52 ± 2.36	15.27 ± 1.95	14.27 ± 2.36	13.62 ± 2.15	13.83 ± 2.21
Control group	53	9.57 ± 2.47	10.59 ± 2.03	11.35 ± 2.04	9.83 ± 2.11	10.25 ± 1.95
*t*		10.549	12.104	6.815	9.159	8.843
*P*		0.001	0.001	0.001	0.001	0.001

**Table 4:** Comparison of incidence of adverse reactions between the two groups [*n* (%)].

Group	*n*	Increased blood glucose	Elevated blood pressure	Pulmonary infection	Infection of digestive canal	Overall incidence
Experimental group	53	1 (1.89%)	0 (0.00%)	1 (1.89%)	1 (1.89%)	5.66% (3/53)
Control group	53	2 (3.77%)	3 (5.66%)	3 (5.66%)	2 (3.77%)	18.87% (10/53)
*χ* ^2^						4.296
*P*						0.038

## Data Availability

The authors confirm that the data supporting the findings of this study are available within the article.
